The article "Exploring the Effect of Dapagliflozin on Alcoholic Kidney Injury and Renal Interstitial Fibrosis in Rats Based on TIMP-1/MMP-24 Pathway" was retracted in 2023. Reasons: unreliable results or conclusions; concerns about the data; concerns about the peer review; concerns about the citations.

# Exploring the Effect of Dapagliflozin on Alcoholic Kidney Injury and Renal Interstitial Fibrosis in Rats Based on TIMP-1/MMP-24 Pathway

**DOI:** 10.1155/2021/6538189

**Published:** 2021-10-21

**Authors:** Yundou Wu, Peijun Song, Xinke Yuan, Dayong Li

**Affiliations:** ^1^Department of Nephrology, The First Hospital of Changsha, Changsha 410005, Hunan, China; ^2^Department of Ophthalmology, The First Hospital of Changsha, Changsha 410005, Hunan, China

## Abstract

**Objective:**

To establish a rat model of alcoholic kidney injury and detect the expression of TIMP-1/MMP-24 in the kidneys of rats with alcoholic kidney injury at the molecular pathological level, so as to explore the mechanism of alcohol abuse leading to kidney injury and renal interstitial fibrosis as well as the alleviation of alcohol-induced kidney injury and inhibition of renal interstitial fibrosis by dapagliflozin.

**Methods:**

48 male rats were randomly divided into 4 groups: control group, alcohol group, alcohol + dapagliflozin group, and alcohol + losartan group, each with 12 rats. Different drugs were administered by gavage for modeling and treatment. Six days later, the rats were sacrificed, blood was collected from the heart to separate the serum, and the blood creatinine (Scr) and urea nitrogen (BUN) contents were detected biochemically. After blood collection, the kidney tissue was taken and fixed in10% neutral formalin. The expression of renal tissue inflammatory factors (CRP, IL-6, and TNF-*α*) and renal fibrosis indexes (LN, HA, and TGF-*β*1) were detected; MMP-24 and TIMP-1 in the kidney tissue of rats in different treatment groups were detected, and Smad3 expression was also detected.

**Results:**

After treatment, the general condition of the alcohol + dapagliflozin group and the alcohol + losartan group improved to different degrees. The weight first decreased and then gradually increased over time. There was no statistical difference in the weight change between the two groups; Compared with the control group, the Scr level, BUN content, renal index, inflammatory factors, and renal fibrosis indexes in the alcohol group were significantly increased (*P* < 0.05); after 6 weeks of treatment, in the alcohol + dapagliflozin group and alcohol + losartan group, Scr level, BUN content, kidney index, inflammatory factors, and renal fibrosis indexes were significantly decreased (*P* < 0.05); the expression of MMP-24 in the kidney tissue of the control group was upregulated, and the expression of TIMP-1 and Smad3 was downregulated; MMP-24 expression was downregulated, and TIMP-1 and Smad3 expression was significantly upregulated (*P* < 0.05) in the rats of the alcohol group. After dapagliflozin and losartan treatment, MMP-24 expression gradually increased and TIMP-1 and Smad3 expression gradually decreased (*P* < 0.05).

**Conclusion:**

Long-term large-scale alcohol intake can cause kidney tissue damage and fibrotic lesions. The expression of fibrotic cytokines such as TIMP-1 and Smad3 will increase, and the expression of MMP-24 will be decreased. However, dapagliflozin and losartan have certain therapeutic effects on the abovementioned lesions. The mechanism may be downregulating TIMP-1 and Smad3 and upregulating the expression of MMP-24 and other cytokines in the kidney.

## 1. Introduction

Alcohol abuse is one of today's important public health problems. Long-term heavy drinking may cause multiple-organ damage. The kidney is an organ of alcohol metabolism and excretion, second only to the liver. Studies have found that alcohol abuse can cause kidney damage, which is mainly characterized by renal tubulointerstitial disease. Common manifestations are renal interstitial edema, inflammatory cell infiltration, and finally, tubular interstitial fibrosis [1]. Excessive deposition of the extracellular matrix (ECM) between the renal tubules and surrounding capillaries destroys the normal microstructure, increases the distance between the capillaries and the renal tubule cells, and damages the capillaries to supply oxygen and nutrients to the renal tubule cells. Injury to renal tubular cells leads to tubular interstitial fibrosis, which in turn affects renal function [2]. The mechanism of renal interstitial fibrosis in alcohol-induced renal injury may be related to the activation of fibroblasts by various factors such as transforming growth factor *β* (TGF-*β*). This research group has examined the expression of transforming growth factor *β*1 (TGF-*β*1) in the kidneys of rats with alcohol-induced kidney injury. Studies have been conducted and the results show that the expression of TGF-*β*1 in rat kidneys is increased [1]. Among all cytokines, TGF-*β* has the strongest fibrotic effect. TGF-*β* reduces the activity of ECM degrading enzymes such as matrix metalloproteinases (MMPs) and increases the activity of degrading enzyme inhibitors such as tissue inhibitors of metalloproteinases (TIMPs), reducing the degradation of ECM leading to renal interstitial fibrosis [2].

MMPs and TIMPs contain a variety of different family members, among which TIMP-1 can combine with activated MMPs to form an enzyme-inhibitor complex, thereby inhibiting the proteolytic activity of MMPs [3]. Studies have shown that the membrane matrix metalloproteinase-24 (MMP-24) plays an important role in the process of degrading the extracellular substance. TIMP-1 overexpression is one of the main causes of renal tubulointerstitial fibrosis, which can cause various abnormal kidney reactions, such as inflammation and immune response, and cooperate with other factors to regulate the proliferation and migration of degenerated fibroblasts. In the process of degeneration, necrosis, and apoptosis, renal interstitial cells are stimulated to secrete cytokines and phagocytes. When phagocytes clear necrotic cells and inhibit cytokines, they will be cleaved by lysosomes to produce elastic fibers and collagen fibers, which will lead to kidney interstitial fibrosis [4, 5]. Signal transducer and activator of transcription (STAT) is a family of transcripts with signal transduction function. The dysregulation of MMPs/TIMPs is also related to the abnormal activation of the STAT pathway, and it plays an important role in the occurrence and development of fibrosis in many organs [5, 6].

Dapagliflozin is a sodium-glucose cotransporter 2 inhibitor (SGLT-2i), a new type of oral hypoglycemic agent. SGLT-2 mediates 90% of the glucose reabsorption in the human body. Dapagliflozin can selectively and strongly inhibit SGLT-2, block the reabsorption of glucose by the proximal convoluted tubules, and reduce blood sugar by increasing the excretion of glucose in the urine. In the rat model of nonalcoholic fatty liver, SGLT-2 inhibitors can significantly increase the activity of STAT3 and improve liver fibrosis [7]. In the rat myocardial infarction model, SGLT-2 inhibitors can significantly increase STAT3 activity, reduce myofibroblast infiltration, and reduce myocardial fibrosis [8]. The above studies suggest that dapagliflozin has renal protective effect and antifibrosis effect, and that it may exert its renal protective effect by interfering with TGF-*β* and MMPs/TIMPs, but the specific mechanism needs to be further studied.

Based on the abovementioned mechanisms of renal injury and renal interstitial fibrosis and the research results of the research group, it is hypothesized that dapagliflozin has the effect of inhibiting alcohol-induced renal injury and reducing renal interstitial fibrosis, possibly by intervening TIMP-1/MMP-24 and so on to play its role in kidney protection. This experiment established a rat model of alcohol-induced kidney injury and used this model to study the expression of TIMP-1/MMP-24 in the alcohol-induced injured kidney of rats and the effect of dapagliflozin on alcohol-induced kidney injury and renal interstitial fibrosis. The results of this study are expected to help us further understand the process of renal interstitial fibrosis and the mechanism of renal protection by dapagliflozin and provide a reference for clinical medication.

## 2. Materials and Methods

### 2.1. Animal Source

Forty-eight healthy 8-week-old Wistar rats, half male and half female, weighing (160±20) g, were purchased from Shanghai Leigen Biological Co., Ltd. The rats were randomly divided into two groups: the control group and the alcohol group. 12 rats were put in the control group and 36 rats in the alcohol group and were reared in separate cages. According to the day and night time course, they were maintained under the conditions of room temperature and stable humidity, with free drinking water and balanced feed.

### 2.2. Experimental Method

#### 2.2.1. Establishment of the Animal Model

After adaptive feeding of 36 rats in the alcohol group, they were fasted every day without water. After 12 hours, they were given normal saline 20 ml/kg and Beijing Erguotou (Baofeng Wine Industry Co., Ltd., production license number: SC11541042100248) diluted to 400 g/L and 8/kg/d, administered three times by gavage. The dose was intragastrically administered once a day. In the same way, the animals in the control group were given the same volume of normal saline by gavage three times a day.

#### 2.2.2. Treatment of Rats in the Alcohol Group

The rats in the alcohol group were divided into three groups: alcohol group, alcohol + dapagliflozin group, and alcohol + losartan group, with 12 rats in each group. Rats in the alcohol + dapagliflozin group were given dapagliflozin (AstraZeneca Pharmaceuticals LP, National Medicine Standard J20170040) 1 mg/kg by gavage, once a day; in the alcohol + losartan group, losartan (Shanghai Yuanye Biological Technology Co., Ltd., Item No.: S80124-1g) 10 mg/kg was given by gavage, once a day. The rats in the alcohol group were given a alcohol 20 ml/kg by gavage.

#### 2.2.3. Specimen Collection

At the end of the 6th week, the rats were weighed and put to death by anesthesia. The chest and abdomen were opened to expose the heart, the heart bag was cut, and a 5 ml syringe was used to insert a needle from the apex of the heart to collect blood. The blood samples were used to measure urea nitrogen and inflammatory factors. Immediately after blood collection, the kidney tissue was weighed and fixed in 10% neutral formalin for later use.

### 2.3. Observation Indicators

#### 2.3.1. General Conditions

The thick and shiny hair of each group of rats, the mental state, the number of activities, and the diet were observed every 10 days, and the weight change was measured.

#### 2.3.2. Renal Function and Kidney Index

The kidney tissues of each group of rats were taken and weighed, and the kidney index (RI) = kidney weight/rat weight was calculated; 0.1 ml of rat blood was added to the reagent tungstate for protein precipitation. The sample was mixed well and centrifuged for 10 minutes, the supernatant was extracted, and then serum creatinine (Scr) level and blood urea nitrogen (BUN) content indicators were tested according to the steps of the kit. The Scr level and BUN content are calculated according to the following formulas: Scr (umol/L) = measured OD value-blank OD value/standard OD value-blank OD value × standard tube concentration (50 umol/L) × 11; BUN content (mmol/L) = measured OD value-blank OD value/standard OD value-blank OD value × standard concentration (10 mmol/L) × the dilution factor of the sample before the test.

#### 2.3.3. Inflammatory Factors and the Progression of Renal Interstitial Fibrosis

The kidney tissue homogenates were prepared, and the enzyme-linked immunosorbent assay (ELISA) was used to detect the expression of the renal tissue inflammatory factors: C-reactive protein (CRP), interleukin-6 (IL-6), and tumor necrosis factor-*α* (TNF-*α*). ELISA was used to detect the content of renal fibrosis indexes in the kidney tissue, including transforming growth factor *β*1 (TGF-*β*1), laminin (LN), and hyaluronic acid (HA).60°C

#### 2.3.4. Expression of MMP-24, TIMP-1, and Smad3 mRNA

The total RNA from the kidney tissue was extracted, and the NCBI gene database was used to obtain the gene sequences encoding MMP-24, TIMP-1, and Smad3 proteins. The primer sequences are shown in Table 1. The PrimeScriptTM RT kit was used to obtain cDNA from each sample, and the PCR reaction solution was prepared according to the SYBR Green one-step PCR kit instructions. The transcription of STAT1, MMP-24, TIMP-1, and Smad3 was detected under the following reaction conditions (94°C for 5 min; 94°C 5 s, 60°C 35 s for 40 cycles), and actin was used as the internal control. The mRNA content of the target gene was quantitatively analyzed with 2^−△△Ct^, and the result was expressed as the value of 2^−△△Ct^ as the mRNA content of the target gene. The fold change in the experimental group relative to the control group was calculated, △△CT(n) = △Ct(n)-△Ct(1), where △Ct(n) = Ct target gene (n)-Ct internal reference gene (n).

#### 2.3.5. Expression of MMP-24, TIMP-1, and Smad3 Protein

The glass plate was cleaned by sodium dodecyl sulfate polyacrylamide gel electrophoresis (SDS-PAGE), dried in an oven, and assembled into the gel maker. Using the following formula, 6.0 ml of 12% separating gel was added, and after the gel had solidified for 40 minutes, 3.0 ml of concentrated gel was added, and the comb was inserted on both sides and allowed to solidify for 40 minutes. The gel maker was put into the electrophoresis tank, which was filled with 1.0% electrophoresis buffer, and the comb was slowly pulled out and loaded with the protein sample and marker. The electrophoresis instrument was used with a constant voltage of 120 V for electrophoresis for 2 hours and waited for the bands to be completely separated. In the past, electrotransfer was placed in 1.0% electrotransfer buffer, and two plates were covered with a sponge and four filter papers. The glass plate was lifted, the required strips were separated, and the PVDF membrane of the corresponding size was cut out. After soaking the PVDF membrane in methanol for about 1 minute, the electrophoresis strips were placed on the filter paper of the black plate, and the PVDF membrane was covered. Here, the air bubbles are removed, the electrotransfer plate is aligned, covered, and placed in the electroporation tank with a constant voltage and a current of 200 mA and the electroporation was performed for 100 min. After the transfer, the membrane was taken out, marked, and placed in 4% blocking buffer on a shaker and blocked for 1.5–2 h. The primary antibody was diluted with 4% blocking special bovine serum blocking solution, and the primary antibody (MMP-24, TIMP-1, and Smad3) was added and incubated overnight at 4°C. The membrane was washed four times with TBST for 15 minutes each time, the horseradish peroxidase-labeled secondary antibody was diluted with 4% blocking special bovine serum blocking solution, and the membrane was washed four times after incubating for 1 to 2 hours at room temperature. Electrochemiluminescence (ECL) was used to develop color (GE Healthcare, USA). After film scanning, the gray value was analyzed with ImageJ software, the ratio of it to *β*-actin was calculated, and the gray value of each histone was detected. The relative quantitative expression of the protein was further analyzed.

### 2.4. Statistical Methods

The results of measurement data were expressed as mean ± standard deviation (*x* ± *s*). If the data conformed to the normal distribution and the variances were uniform, one-way ANOVA was used for the comparison of means between groups and the LSD multiple test was used for pairwise comparisons between groups. The Kruskal–Wallis H test was used for those who do not conform to the normal distribution or if the variance was not uniform. SPSS 22.0 statistical software was used to analyze the experimental data. *P* < 0.05 indicates that the difference is statistically significant.

## 3. Results

### 3.1. General Observation

During the establishment of the model, the control group had thick hair, bright lustre, good spirits, frequent activities, normal diet, and weight gain over time; the alcohol group had dull hair, patchy hair falling, poor spirits, lack of energy, significantly reduced diet, and the weight first decreasing and then slowly increasing (*P* < 0.05). After treatment, in the alcohol + dapagliflozin group and the alcohol + losartan group, the hair color, shedding, food intake, reaction sensitivity, etc. of the rats were improved to varying degrees. The body weight first decreased and then gradually increased over time (*P* < 0.05). There was no statistical difference in weight change between the two groups (*P* > 0.05), as shown in Figure 1.

### 3.2. Scr Level, BUN Content, and Kidney Index of Rats

After modeling, compared with the control group, Scr level, BUN content, and kidney index in the alcohol group were significantly increased and the difference was statistically significant (*P* < 0.05); as shown in Figures 2(a) and 2(b); after 6 weeks of treatment, the Scr level, BUN content, and renal index in the alcohol + dapagliflozin group and alcohol + losartan group were significantly lower as compared with the alcohol group *P* < 0.05.

### 3.3. Inflammation of the Kidney Tissue in Rats

The results showed that compared with the control group, the inflammatory factors CRP, IL-6, and TNF-*α* in the alcohol group were significantly increased and the difference was statistically significant (*P* < 0.05); after 6 weeks of treatment, CRP, IL-6, and TNF-*α* were lower in the alcohol + dapagliflozin group and the alcohol + Losartan group than in the alcohol group (*P* < 0.05). There was no statistical difference between the alcohol + dapagliflozin group and the alcohol + Losartan group (*P* > 0.05), as shown in Figure 3.

### 3.4. Progression of Renal Interstitial Fibrosis in Rats

The results showed that compared with the control group, the renal fibrosis indexes TGF-*β*1, LN, and HA were significantly increased in the alcohol group and the difference was statistically significant (*P* < 0.05); after 6 weeks of treatment, the alcohol + dapagliflozin group and the alcohol + losartan group had lower TGF-*β*1, LN, and HA (*P* < 0.05) than the alcohol group. There was no statistical difference between the alcohol + dapagliflozin group and the alcohol + losartan group (*P* > 0.05), as shown in Figure 4.

### 3.5. Expression of MMP-24, TIMP-1, and Smad3 mRNA in the Kidney Tissue

qRT-PCR detected the expression of MMP-24, TIMP-1, and Smad3 mRNA in the kidney tissue, and compared with the control group, the MMP-24 mRNA in the kidney tissue of the alcohol group decreased and the expression of TIMP-1 and Smad3 mRNA were significantly increased. The difference was statistically significant (*P* < 0.05); after 6 weeks of treatment, compared with the alcohol group, the MMP-24 mRNA in the kidney tissue increased, and the expression of TIMP-1 and Smad3 mRNA decreased(*P* < 0.05) in the alcohol + dapagliflozin group and the alcohol + losartan group and there was no statistical difference between the alcohol + dapagliflozin group and the alcohol + losartan group (*P* > 0.05), as shown in Figure 5.

### 3.6. Expression of MMP-24, TIMP-1, and Smad3 Protein in the Kidney Tissue

WB detected the expression of MMP-24, TIMP-1, and Smad3 protein in the kidney tissue. Compared with the control group, the MMP-24 protein in the kidney tissue of the alcohol group decreased and the expression of TIMP-1 and Smad3 protein was significantly increased. The difference was statistically significant (*P* < 0.05); After 6 weeks of treatment, compared with the alcohol group, the MMP-24 protein in the kidney tissue increased, and the expression of TIMP-1 and Smad3 protein decreased (*P* < 0.05) in the alcohol + dapagliflozin group and the alcohol + losartan group and there was no statistical difference between the alcohol + dapagliflozin group and the alcohol + losartan group (*P* > 0.05), as shown in Figure 6.

## 4. Discussion

Alcohol abuse is a major social public health problem. It causes damage to multiple organs such as the liver, brain, and stomach. The damage is the most obvious [9, 10]. Its metabolites have damaging effects on multiple organs of the whole body. In addition, the imbalance of nutrition ratio caused by long-term alcohol intake is also one of the causes of damage [11]. Alcohol-induced damage to the body can be divided into acute and chronic. Acute kidney damage can lead to organ failure and death. Chronic kidney damage (CKD) mainly affects renal function and pathology of renal tubules, glomeruli, and renal interstitial structures and sexual change. After alcohol enters the body, it is mainly metabolized by the liver, and 10%–15% can be metabolized by the kidneys. And, the metabolites of alcohol such as acetaldehyde and butyric acid can also stimulate the body's unbalanced regulation of aldosterone and angiotensin [12], increase kidney load, gradually change the structure of kidney tissue, and further aggravate the damage of kidney function.

The metabolism time of alcohol in rats is 8–24 hours. Alcohol is mainly metabolized by the liver, the kidney can directly metabolize part of the alcohol first, and then most of the secondary alcohol metabolites such as acetaldehyde and butyric acid are also metabolized by the kidney. Alcohol itself or its primary metabolites has toxic effects on the kidneys [13]. In addition, the results of this experiment showed that the alcohol group was found to be in poor general condition after 6 weeks of model establishment and the renal function indexes, BUN content, and SCr levels were high, which is consistent with recent domestic and foreign reports [14–16] and previous studies on alcoholic kidney injury in this research group, confirming the high reliability of the modeling method in this study. The reason for the poor general condition of the alcohol group may be due to gavage injury, esophageal bleeding or alcoholic stomach injury, and gastric bleeding. In the early stage, rats have large changes in body weight and poor adaptability to alcohol. In the later stage, the range of weight changes decreases and it causes lethargy, weakness, and increased lacrimal secretions. It may be that alcohol has inhibitory effects on the sensory and motor nerve centers of rats. The reason for the high levels of renal function indicators BUN and SCr may be due to the reabsorption capacity and the reduction of glomerular filtration rate caused by the damage of the renal tubules [17].

In the examination of the kidney tissue of rats in the alcohol group, we also found that the inflammation of the kidney tissue and the progress of renal fibrosis are high, which may be due to chronic alcohol consumption causing renal interstitial fibrosis to be affected by oxidative stress and inflammatory regulation [18]. More and more pieces of evidence show that the stress and inflammatory cytokines produced by the oxidation of reactive oxygen species are very important in renal tubular cell proliferation and renal fibrosis [19–21]. Moreover, the TGF-*β* family is closely related to a variety of chronic renal fibrosis. However, it is now believed that the pro/antifibrotic effect of the TGF-*β* superfamily is mainly achieved by activating its intracellular signal transduction protein Smad family. The Smad gene family is an important intracellular regulatory molecule in the TGF-*β* signal transduction pathway. Among all the cytokines, TGF-*β* has the strongest fibrosis effect and LN and HA are related to the degree of fibrosis. And some studies have shown [22] that TGF-*β* affects the activity of MMPs and TIMPs and reduces the degradation of ECM and leads to renal interstitial fibrosis. In our study, it was also found that MMP-24 was decreased in the kidney tissue and the expression of TIMP-1 and Smad3 proteins were significantly increased, suggesting that the expressions of MMP-24, TIMP-1, and Smad3 are related to alcohol-induced kidney injury and the degree of renal fibrosis.

Studies have shown that dapagliflozin has an independent renal protective effect, which can improve renal hypoxia and reduce renal inflammation without relying on its hypoglycemic effect [23]. At the same time, dapagliflozin also has an antifibrosis effect. This study will also use losartan as a control group. Losartan is an angiotensin II-I receptor antagonist (AT1RA). Angiotensin II can promote renal fibrosis by activating the TGF-*β*1/Smad3 pathway [24]. In addition to affecting the renin-angiotensin system, losartan can also have an antifibrotic effect by affecting a variety of cytokines. The renal protection and antifibrosis effects of losartan have been confirmed by a number of studies [24–26]. The results of this study found that the general condition and weight gain of rats treated with dapagliflozin and losartan were better than those in the alcohol group. The Scr level, BUN content, and kidney index all showed a significant downward trend, and the degree of inflammation invasion and progression of renal fibrosis decreased. The expression of MMP-24, TIMP-1, and Smad3 in kidney tissues was detected. Compared with the alcohol group, the alcohol + dapagliflozin group and the alcohol + losartan group had higher levels of MMP-24 mRNA and protein in the kidney tissue and TIMP -1 and Smad3 expression of mRNA and protein decreased, suggesting that dapagliflozin has a protective effect on the kidney tissue of alcohol-induced kidney injury rats and can reduce renal tissue inflammation and renal fiber progression, upregulate MMP-24, and downregulate TIMP-1 and Smad3; its effect is similar to the therapeutic effect of losartan on damaged tissues.

In summary, long-term excessive alcohol intake can cause kidney tissue damage and fibrotic lesions. The expression of fibrotic cytokines such as TIMP-1 and Smad3 will increase, and the expression of MMP-24 will decrease, while dapagliflozin and losartan have a certain therapeutic effect on the abovementioned lesions It has a certain therapeutic effect on the abovementioned lesions. The mechanism may be downregulating TIMP-1 and Smad3 and upregulating the expression of MMP-24 and other cytokines in the kidney.

## Figures and Tables

**Figure 1:** Changes in body weight of rats in each group. Note: compared with the control group, ^*∗*^*P* < 0.05; compared with the alcohol group, ^#^*P* < 0.05.

**Figure 2:** Rat Scr level, BUN content, and kidney index. Note: compared with the control group, ^*∗*^*P* < 0.05; compared with the alcohol group, ^#^*P* < 0.05.

**Figure 3:** Inflammation of the kidney tissue in rats. Note: compared with the control group, ^*∗*^*P* < 0.05; compared with the alcohol group, ^#^*P* < 0.05.

**Figure 4:** The progression of renal interstitial fibrosis in rats. Note: compared with the control group, ^*∗*^*P* < 0.05; compared with the alcohol group, ^#^*P* < 0.05.

**Figure 5:** Expression of MMP-24, TIMP-1, and Smad3 mRNA in the kidney tissue. Note: compared with the control group, ^*∗*^*P* < 0.05; compared with the alcohol group, ^#^*P* < 0.05.

**Figure 6:** Expression of MMP-24, TIMP-1, and Smad3 protein in the kidney tissue. Note: compared with the control group, ^*∗*^*P* < 0.05; compared with the alcohol group, ^#^*P* < 0.05.

**Table 1:** qRT-PCR primers.

Primer sequence	Forward (5'–3')	Reverse (5'–3')
MMP-24	CGAGCTATCCACTCATCAAACA	TGAACCATAACGCACAGACC
TIMP-1	CCCAGAACCGCAGTGAAG	GTGGCAGGCAAGCAAAGT
Smad3	ACTACAGCCATTCCATCCC	TAGGTTTGGAGAACCTGCG
*β*-Actin	CAATAGTGATGACCTGGCCGT	AGAGGGAAATCGTGCGTGAC

## Data Availability

The data used and analyzed during the current study are available from the corresponding author on reasonable request.
